# Exploring the Ability to Perform Activities of Daily Living and Cognitive Status after Hospitalization with COVID-19: A Multiple Case Study

**DOI:** 10.1155/2022/4605989

**Published:** 2022-03-29

**Authors:** Kate Allen Christensen, Jan Christensen, Signe Janum Eskildsen

**Affiliations:** Department of Occupational Therapy and Physiotherapy, Copenhagen University Hospital, Rigshospitalet, Copenhagen, Denmark

## Abstract

**Background:**

Multidisciplinary rehabilitation including occupational therapy after COVID-19 is recommended. However, evidence on how COVID-19 affects the ability to perform activities of daily living (ADL) is sparse.

**Objective:**

The aim of this study was to explore the ability to perform ADL and cognitive status in patients with COVID-19 at time of discharge and three months postdischarge.

**Methods:**

This prospective multiple case study included adults with COVID-19, who at time of discharge had decreased ADL performance compared to habitual functional level. Data collection included Assessment of Motor and Process Skills (AMPS) and Montreal Cognitive Assessment (MoCA) at discharge and three-month follow-up. Exploratory analysis was used to identify similarities and trends within and across cases.

**Results:**

Eleven patients were included. 75% had a significant increase in motor ability measures, and 27% had a significant increase in process ability measures at follow-up. 67% of follow-up cases showed mild cognitive impairment, where executive functioning and memory were most predominant.

**Conclusions:**

The ability to perform ADL was affected at discharge and at three-month follow-up. Furthermore, mild cognitive impairment was present at both hospital discharge and follow-up in most cases. *Significance*. Occupational therapists can apply performance-based assessments to identify the need for rehabilitation of ADL in patients with COVID-19 during and posthospitalization.

## 1. Introduction

The coronavirus disease 2019 (COVID-19) global pandemic has resulted in over 200 million confirmed cases and over four million reported deaths worldwide [1]. The clinical presentation of COVID-19 can vary from asymptomatic to severe illness and acute respiratory failure ultimately requiring mechanical ventilation and intensive care treatment and/or leading to possible death. Studies describe a variety of sequalae regardless of the severity of the initial clinical presentation including fatigue, breathlessness, fever, headache, muscle weakness, gastrointestinal symptoms, loss of taste and smell, anxiety, depression, and cognitive symptoms [2–11]. Cognitive symptoms include affected memory, concentration, and executive functioning [4, 6, 8]. For patients with COVID-19, physical complaints may be prominent in the acute phase during intensive care unit (ICU) admission, while cognitive and mental symptoms manifest later, especially when patients return to the domains of everyday life such as work, spare time interests, and family roles [7, 12]. Even individuals with COVID-19 who were not hospitalized describe the need for rehabilitation of fatigue and cognitive symptoms as well as difficulty returning to usual activities [4, 8, 9, 12–14]. Symptoms can have diverse effects on the functional abilities of individuals and multidisciplinary rehabilitation after COVID-19 is recommend, and this includes occupational therapy (OT) [8, 13, 15]. Researchers recommend OT assessments of occupational performance for COVID-19 patients to identify rehabilitation needs of activity, occupational performance, and participation including cognitive disabilities [16, 17].

Recently, two single-case reports describing OT evaluation and treatment approaches for a client with COVID-19 have emerged [12, 14]. Both report the possible distinct role of OT to this patient group where physical, cognitive, psychological, and emotional symptoms affected their ability to perform usual ADL. Regardless of inpatient or outpatient settings, OT focused on activity engagement, fatigue management, and cognitive strategies with the goal of returning to usual everyday life [12, 14].

We did not have guidelines for OT practice when patients with COVID-19 were initially referred to OT at Copenhagen University Hospital, Rigshospitalet (RH), Denmark. Thus emerged, the need for gaining knowledge and evidence of patients' abilities to participate in ADL, their cognitive status and rehabilitation needs.

The aim of this study was to explore similarities and trends in ability to perform ADL and cognitive status at discharge and three months postdischarge in patients diagnosed with COVID-19, who at discharge had diminished ADL performance compared to habitual functional level. Furthermore, we aimed to explore rehabilitation needs and the implications for OT practice.

## 2. Material and Methods

### 2.1. Study Design

A prospective multiple case study design was chosen [18]. This design makes it possible to follow a novel and heterogenic group of patients with the same diagnosis, perform analysis within and across cases, and generate hypothesis for further research [18–20]. Source of data includes electronic patient records and assessments at hospital discharge and at three-month postdischarge by trained occupational therapists. The reporting of this study follows the guideline of Strengthening the Reporting of Observational studies in Epidemiology (STROBE) [21].

### 2.2. Study Setting

All cases were enrolled from RH, a highly specialized hospital where medical care is provided in an up-front tax paid public healthcare system. Patients can be referred to the OT department from all other departments when the need for rehabilitation is identified. In-patient rehabilitation is initially provided by occupational therapists during hospital admission. Upon discharge, a physician, in collaboration with a multidisciplinary team, is responsible for assessment of rehabilitation needs of patients and where relevant complete a *rehabilitation plan* as referral for further community rehabilitation [22]. During the COVID-19 pandemic, multidisciplinary treatments were gradually adjusted and improved as clinical work experience was obtained. Initially, there were few referrals to OT, but as the patients with COVID-19 survived their acute treatment or ICU admission, they began to present with symptoms of dysphagia and decreased ability to perform ADL, fatigue, and neurological impairments.

The organization of departments treating patients with COVID-19 varied across the data collection period. During periods with increased COVID-19 hospitalization (spring 2020 and winter 2020-2021), cohort isolation wards specific for COVID-19 patients were established. During periods with less COVID-19 admissions, the patients were admitted to general wards, including the wards of the Department of Infectious Diseases. Cases were recruited from the cohort isolation wards as well as wards on the Department of Infectious Diseases between May 2020 and January 2021.

### 2.3. Data Collection

Data collection included Assessment of Motor and Process Skills (AMPS) [23, 24] as well as Montreal Cognitive Assessment (MoCA) [25] at hospital discharge and at three-month follow-up. At hospital discharge, AMPS and MoCA were performed by AMPS-calibrated occupational therapists. At follow-up, AMPS-calibrated occupational therapists and MoCA by experienced occupational therapists or a neurologist as part of a concurrent COVID-19 project. All occupational therapist involved in this study were authorized and registered in Denmark. Recruitment was conducted by four occupational therapists, that provided treatment for patients with COVID-19. These occupational therapists had three to five years of experience in varying hospital wards and patient categories and specific experience in rehabilitation, though primarily with neurological patients. As COVID-19 was a novel illness at the time of inclusion, experience with this specific patient group was sparse.

The first author called patients four weeks prior to the three-month follow-up to confirm participation and plan activities for AMPS. After case 1 declined follow-up due to low functional level and lengthy transportation to the hospital, a collaboration with occupational therapists in the community was initiated. If participants declined to participate in the follow-up due to lengthy transportation, the first author, with permission of the patient, contacted the multidisciplinary community rehabilitation units to ask the local occupational therapists if they could perform follow-up testing. The three community occupational therapists who were contacted accepted.

### 2.4. Participants

Patients were included if they were diagnosed with COVID-19, admitted to RH and at discharge had lower ability to perform ADL compared with abilities prehospitalization. For example, if the patients needed assistance in activities like toileting, bathing, or dressing, which they would usually perform independently at home, patients were considered eligible for inclusion if they were adults ≥ 18 years and able to understand and follow instructions in Danish during testing. Patients were excluded if they were in isolation and sufficiently challenging ADL tasks could not be performed on the ward due to the COVID-19 restrictions, e.g., if the task required observation of kitchen activities.

Information of changes in ADL ability was primarily obtained through the OT intervention via interview and/or observation of the patient. Three cases were identified during multidisciplinary conferences where clinical handover by nurses and physiotherapists reviled ability discrepancies in current and prior hospitalization ADL performance.

### 2.5. Data Sources

AMPS was used to investigate and describe ability to perform ADL [23, 24], and MoCA was used to investigate and describe cognitive function [25]. Information on rehabilitation needs and demographic variables were obtained from electronic patient records. AMPS is an OT-specific observational assessment of motor and process skills during activity performance. AMPS can evaluate the ability to perform instrumental and personal ADL and document change over time [24]. Instrumental ADL includes activities such as cooking, shopping, or housework required for independent living. Personal ADL are related to self-care such as washing and dressing [24]. AMPS provides information about the quality of the patients' performance in terms of *effort*, *efficiency*, *safety*, and *independence* [23]. This observational assessment is standardized and tested on more than 100.000 persons internationally [24]; however, to our knowledge, no academic literature has used AMPS for COVID-19 patients. It has test-retest and interrater reliability and validity when used among various populations [24].

In collaboration, the patient and occupational therapist choose two ADL tasks, that the patient wants or needs to perform and find challenging. The patient performs the two tasks after standardized instruction by the occupational therapist. The quality of 16 ADL motor skills (e.g., body position, obtaining and holding objects, and sustaining performance) and 20 ADL process skills (e.g., applying knowledge, organizing space and objects, and adapting performance) are scored by a calibrated assessor on a 4-point ordinal scale. The scores of the 16 motor and 20 process skills are analyzed using the Rasch-based computer AMPS-software (Occupational Therapy Assessment Package (OTAP), Center for Innovative OT Solutions, Fort Collins, Colorado, USA), which converts raw skill scores into logistically transformed probability units (logits), that are presented in two graphic rapports of ADL motor and ADL process skills. The logits are adjusted for rater severity and difficulty of the ADL tasks observed. Both rapports reflect *safety* and *independence*. The motor ability measure indicates how much *effort* (clumsiness and/or increased physical effort or fatigue) the patient experiences during performance of ADL, and the process ability measure how *efficient* (inefficiency and/or disorganization) the patient is during performance [23, 24, 26]. A bold text on the graphic rapports describes the overall quality of ADL task performance commonly observed by people with the same ADL ability measure, e.g., *questionable*, *mild*, *moderate*, or *marked* clumsiness and/or increased physical effort or fatigue or inefficiency and/or disorganization.

A motor skill logit of 2.0 is a criterion referenced cut-off, where a person is likely to begin showing slight clumsiness or physical effort. There is a risk zone of 0.3 logits, and logits ≥ 2.3 reflect skilled (no clumsiness or effort), safe, and independent ADL task performance. The cut-off for process skills is 1.0 logit, where a person is likely to begin showing inefficiency, and logits ≥ 1.3 reflect *efficient* (timely and spatially organized), safe, and independent ADL task performance [24].

MoCA is a cognitive screening tool. A one-page, 30-point, pen, and paper assessment administered by clinicians in approximately 10 minutes [25]. The screening tool covers the cognitive domains: attention, visuospatial abilities, executive functioning, memory, language, and orientation. Attention is tested through three tasks: auditory motor attention (1 point), serial subtraction (3 points), and memorizing number range (2 points). Visuospatial abilities are tested in two tasks: copy of a cube (1 point) and clock drawing (3 points). Executive functioning through a trail making task (1 point), phonemic fluency (1 point), and a two-item abstraction task (2 points). Memory through delayed recall of five words (5 points). Language uses a three-item naming task (3 points) and repetition of two complex sentences (2 points): orientation to date, month, year, day, place, and town (6 points). MoCA scores range between 0 and 30, a higher score indicating higher cognitive functioning. The score is education-corrected by giving an additional point to persons with ≤12 years of education. Based on research in various populations, MoCA is found to have an adequate concurrent validity with comprehensive cognitive measurements for cognitive deficits, has excellent test-retest reliability, and is sensitive in detecting mild cognitive impairment [25, 27, 28]. MoCA has been used in studies of patients with COVID-19 [10, 29, 30]. The Danish version of MoCA was used in this study [31]. A summary MoCA score of <26 is used as a cut-off in detecting mild cognitive impairment [25].

### 2.6. Data Analysis

Inspired by Yin [18], we allowed for exploratory analysis of the data to identify similarities, trends, and patterns of ADL performance, cognitive status, rehabilitation needs, and implications for OT within and across cases. A matrix of variables across cases structured the gathered information. Some variables were predefined for each participant, e.g., age, sex, days to discharge test, ICU admission, AMPS, and MoCA results. Other variables like reason for referral, OT treatment goals, and plans emerged, through an iterative process of going through data several times [18]. Similarities and trends among cases and variables were discussed between all authors at several meetings [18, 20].

Case descriptions, as well as data on non-participators, will be presented in text and tabular forms presenting median, as well as range for continuous data, frequencies, and percentages for all categorical and dichotomized data.

The data presentation for each individual case includes the performed AMPS tasks and difficulty, AMPS results in logits, AMPS age and sex adjusted percentile rank, and the MoCA results.

When interpreting AMPS at follow-up, a higher logit for the second observation indicates improved ADL ability. The ADL motor ability measures must differ by at least 0.5 and/or the ADL process ability measures by at least 0.4 to indicate that the assessed person's ADL ability has a high likelihood to have changed significantly between two AMPS observations [24]. It is not recommended to evaluate AMPS raw score in terms of effect [24]. However, the raw scores can be highly relevant in guiding OT recommendations and will be presented as raw data.

Trends across MoCA domain scores will be presented, and trends between AMPS process logits and MoCA total score will be analyzed. Individual scores, logits, and changes over time between discharge and three-month follow-up will be presented visually using a spaghetti plot for both AMPS and MoCA.

### 2.7. Ethics

The study complied with ethical principles for medical research as described in the Helsinki Declaration [32]. Eligible patients received oral and written information about the study by the occupational therapist, and if willing to participate in the study, the patient signed an informed consent. Patients who declined to participate were asked whether their age, sex, and length of stay in ICU, and reason not to participate could be documented. The Danish data protection agency approved the handling of data (P-2020-499).

## 3. Results

Fourteen patients were assessed for eligibility, and eleven patients were included in this study. A flow diagram in Figure 1 illustrates inclusions, data collection, missing data, and participants included for analyses. The three nonparticipators declined due to low mental and/or physical energy. Low mental and/or physical energy was prevalent in all cases. No specific differences or patterns were identified between participators and nonparticipators in terms of age, gender, and ICU admissions. Nine of the participants were admitted with COVID-19 as their primary diagnosis. Seven were in ICU with a median stay of 24 days (range 10 to 80). The length of stay in hospital from admission to discharge assessment ranged from seven to 90 days with a median of 20 days. Eight patients were referred to OT, seven referrals for assessment of swallowing abilities and one referral for ADL assessment before discharge. Participant characteristics are presented in Table 1.

Six of the seven cases referred with dysphagia had been admitted to the ICU. The OT interventions ranged from reassessment of swallowing, eating and drinking, and assessment of ADL which involved the facilitation to participate in personal ADL such as washing the face and lifting a glass to the mouth, as well as more complex activities of showering and dressing. Full case descriptions are presented in Table 2.

At discharge assessment, nine participants completed AMPS and MoCA the same day. Due to fatigue, two patients asked to be tested on separate days with one and four days apart (cases 4 and 8). Due to general weakness and geographical distance, it was not possible to complete follow-up assessments at the hospital in four cases (cases 1, 3, 6, and 7). In three of these cases, follow-up assessments were conducted by an occupational therapist in the local community (cases 3, 6, and 7).

Follow-up AMPS were performed on eight participants (73%): follow-up MoCA on six participants (55%). The AMPS three-month follow-up assessments were conducted with a median of +1.5 day (range -15 to +25 days), to the exact day, where three months had passed since discharge testing. One participant declined MoCA due to rehospitalization (case 8), however, participated in an AMPS during standard OT intervention during rehospitalization at the scheduled time for follow-up. Five of the MoCA follow-up assessments were performed on the same day as AMPS, and one was performed 60 days later (case 3). No trends were identified in loss to follow-up and lower or higher test results at discharge.

### 3.1. Ability to Perform ADL

Table 3 sums up the difficulty level of AMPS activities at discharge and follow-up. The majority of AMPS activities chosen by the patients as difficult to carry out at discharge were classified as ≤ “easier than average ADL tasks.” This included patients that prior to admission had been independent in all ADL, including work. The patients able to complete ≥ “average ADL tasks” at follow-up were the patients whom prior to admission had been independent in all ADL or at least personal ADL.  Table 4 depicts the individual difficulty of AMPS activities for each case, the AMPS motor, and process ability measures in logits.

#### 3.1.1. Motor Ability Measures

Analysis for trends in the data from AMPS showed that at discharge, all cases had a motor ability measure below the cut-off of the criterion referenced 2.0 logits, ranging from -1.3 logits (marked) to 1.9 logits (questionable to mild), indicating clumsiness and/or increased physical effort or fatigue during ADL task performance, see Figure 2.

At follow-up, all cases had improved motor ability measures with a median change of 1.1 logits (range 0.1 to 1.5). Six cases (75%) showed significant improvements, with increased logits by at least 0.5 (cases 2, 3, 4, 5, 6, and 7).

#### 3.1.2. Process Ability Measure

Contrary to the trends of motor ability measures, trends and patterns across process ability measures showed greater variation between patients at both discharge and follow-up (see Figure 3). At discharge assessment, nine cases (82%) had a process ability measure below (or just above) the criterion referenced cut-off of 1.0 logit ranging from 0.0 to 1.2 logits, indicating (questionable) inefficiency and/or disorganization during ADL task performance.

At follow-up, seven cases (88%) had improved process ability measures, the median change being 0.25 logits (range -0.4 to 0.9), but only three (38%) showing significant changes with process ability measures improving by at least 0.4 logit (cases 3, 4, and 7). Cases 4, 7, and 8 displayed efficient process ability measures during ADL task performance at follow-up.

#### 3.1.3. Motor and Process Performance Skills at Hospital Discharge

At discharge testing, occupational therapists reported similar predominant problematic motor performance skills (raw scores) across cases in the electronic patient journals. In 10 out of 11 cases, the motor performance skill, *endures*, was reported as problematic, and nine cases had especially difficulty in *reaches. Flows* was described in six cases and *grips* in five. No patterns nor similarities were found across cases in the process performance skills (raw scores) highlighted as predominant.

### 3.2. Trends and Similarities in Significant Changes in Ability to Perform ADL

When searching for patterns across significant changes in AMPS results between discharge and follow-up, two groups were identified: one group of three patients (27%) with significant changes in both *motor* and *process* ability measures and another group of three patients (27%) showing significant change in *motor* ability measures only.

#### 3.2.1. Significant Changes in Motor and Process Ability Measures (Cases 3, 4 and 7)

The AMPS result of cases 3, 4, and 7 indicated that their ability to perform ADL had a high likelihood to have changed significantly in both *motor* and *process* ability measures. When comparing all cases, exploratory analysis showed similarities across these three cases. All three cases had been referred to OT during admission and were all discharged to inpatient community rehabilitation units. These were the only participants to complete follow-up, whom at discharge testing had motor ability measures indicating *marked or moderate-marked* clumsiness and/or increased physical effort or fatigue during ADL task performance.

Two of the three cases (cases 3 and 7) needed assistance for personal ADL prior to admission and had several coexisting illnesses. These two patients did not have the energy levels to attend the follow-up assessment at the hospital, and these were conducted in a community rehabilitation facility. As illustrated in Figure 2, all three patients were still below the criterion-referenced cut-off of 2.0 logits in motor ability measures indicating *mild to moderate* clumsiness and/or increased physical effort or fatigue during ADL task performance at follow-up. In contrast, two of the patients showed process ability measures of efficient (timely and spatially organized) ADL task performance at follow-up (cases 4 and 7 in Figure 3).

#### 3.2.2. Significant Changes in Motor Ability Measure Only (Cases 2, 5, and 6)

Three cases (cases 2, 5, and 6) had significant changes in ADL *motor* ability measures at follow-up. Their *process* ability measures did not show significant change. When looking for trends, patterns, and similarities across these cases, all were independent prior to admission; two were employed (case 2 and 5). All three cases had process ability measures at cut-off or in the risk zone, where questionable inefficiency or disorganization during ADL task performance could be observed at discharge as well as follow-up. At follow-up, AMPS age and sex adjusted percentile rank indicated that 90.5% of healthy people of the same age likely had a higher ADL process ability measure. At follow-up, case 5 had started work part time, and case 2 was able to carry out personal ADL but not complex ADL like heavy household or work. Case 6 was retired, and she felt close to habitual functional level, although did experience fatigue. Cases 5 and 6 were not referred to OT during admission.

Cases 5 and 6 were the only cases, of all, showing skilled (no clumsiness or effort), safe, and independent motor abilities during ADL task performance at follow-up with motor logits above 2.3.

As presented in Table 4 and illustrated in Figure 4, all three cases had an improvement or had the same score in MoCA at follow-up. Case 2 showed a notably improved MoCA score from 18 to 28.

### 3.3. Cognitive Status

At discharge, the median total MoCA score was 24 (range 8-30). Eight cases (73%) had a total MoCA score indicating mild cognitive impairment with a cut-off of <26. The median of the six follow-up MoCA scores (cases 2, 3, 5, 6, 7, and 11) was 24.5 (range 21-30); the MoCA score of four follow-up cases (67%) indicated mild cognitive impairment with <26. Trends across cases were an increase in MoCA score between discharge and follow-up: a tendency to high scores in *orientation* in time and place, with 73% of cases achieving the highest score at discharge and 83% at follow-up. Furthermore, *memory* and *executive functioning* appeared to be the dominant domains most difficult across cases.  Table 5 depicts domain scores at discharge and follow-up.

#### 3.3.1. Independence Preadmission and Cognitive Status

Across cases, it was found that for the patients independent in ADL prior to admission (cases 2, 4, 5, 6, 8, and 10), 50% had a total MoCA score indicating normal cognitive functioning at discharge (cases 4, 6, and 8). The three other cases were below cut-off <26 (cases 2, 5, and 10). Cases 2, 5, and 6 completed follow-up MoCA: two having MoCA total scores ≥ 26; case 5 remained <26 indicating mild cognitive impairment.

#### 3.3.2. Need of Assistance Preadmission and Cognitive Status

Of the cases, whom at habitual functional level needed assistance for personal or instrumental ADL (cases 1, 3, 7, 9, and 11), all had a MoCA score below 26. We were not able to find similarities in MoCA scores at discharge among the groups of cases needing help for personal ADL (cases 1, 3, and 7) and cases needing help for instrumental ADL only (cases 9 and 11).

### 3.4. Patterns in AMPS and MoCA Scores

Across all cases, no pattern could be found between the MoCA results and AMPS results. For example, the three cases showing significant changes in motor ability measures (cases 2, 5, and 6) had very similar process ability measures, however, very different MoCA scores. Likewise, case 7 showed a rise in efficient process ability measures at three-month follow-up, but at the same time having a fall in MoCA from 24/30 to 21/30 at follow-up. Unfortunately, the MoCA of case 4 is missing at follow-up and therefore trends between MoCA and an efficient process ability measure that are not possible to comment on.

### 3.5. Rehabilitation Needs

All cases received a multidisciplinary rehabilitation plan at discharge from hospital for further rehabilitation in the community. Occupational therapists participated in the completion of 10 rehabilitation plans. The rehabilitation plans all described further need for facilitation of independence in habitual ADL level, including return to work and complex instrumental daily activities, where it was relevant. They also focused on fatigue and endurance during activity performance, some specifically naming the use of principles of energy conservations. Examples included education in adapting activity performance and/or the environment to be able to carry out ADL. The majority of rehabilitation plans described a need for an increase in global muscle strength. Only few rehabilitation plans mentioned the need for further swallowing assessments and/or treatment. (cases 2 and 9) (Table 2).

## 4. Discussion

### 4.1. Summary of Findings

Eleven patients with COVID-19 and decreased ADL performance at hospital discharge were included in this study. Three-month follow-up included AMPS data from eight cases and MoCA data from six cases. The cases represented a diverse sample across age, sex, preexisting illness, and habitual functional level; some needing assistance in ADL prehospitalization, and some working full time and/or being independent in all ADL. The course of admission was heterogenic in terms of length of stay, ICU treatment, and referrals for OT. Across cases, very similar P-ADL tasks were performed at discharge, no matter the prior level of functional ability. At follow-up, the difficulty of ADL tasks performed varied, where cases being independent prehospitalization performed more challenging ADL tasks.

Ability to perform ADL was affected at discharge as well as three-month postdischarge across all cases. This included the following: low endurance and a trend of low motor ability measures; all cases being below the criterion referenced cut-off at discharge and all cases showing increased motor skills during ADL task performance with 75% of cases having a *significant* increase in motor ability measures. Furthermore, most cases still showed signs of clumsiness and/or increased physical effort or fatigue at follow-up. In contrast, the cases showed larger variation in process ability measures. Only 27% had a *significant* increase in process ability measures at follow-up, and no patterns were identified across process skills. Three of the cases habitually independent in ADL (50%) did not have significant changes in process ability measures at three-month follow-up. This revealed questionable inefficiency or disorganization during ADL task performance. We could not find any patterns across cases between MoCA and AMPS scores.

Mild cognitive impairment was detected in the majority of cases at discharge (73%). Executive functioning and memory appeared the most difficult across cases and orientation the least difficult. Attention and memory scores showed a diverse heterogenic pattern at follow-up, e.g., some scores being lower at follow-up, than discharge. Four out of the six follow-up cases had mild cognitive impairment, including one case, who had returned to work part time.

Interestingly, the majority of patients with COVID-19 referred to OT were referred for assessment of dysphagia, but only two still needed rehabilitation for dysphagia after hospital discharge. Rehabilitation needs postdischarge focused on interventions regarding endurance, low mental/physical energy, and performing ADL, more specifically focusing on motor skills and for some, also on process and cognitive skills.

Currently, no other research using AMPS for assessing ADL performance in patients with COVID-19 has been identified. In a study from the United Kingdom in 2020 [9], 100 patients with COVID-19 were telephone interviewed a mean of 48 days after discharge from a hospital to identify postdischarge symptoms and rehabilitation needs. One third of these patients required ICU treatment and hospital length of stay ranged from four to 16 days. Similar to our findings, patients identified endurance problems, which was categorized as fatigue as well as disabilities in mobility, self-care, and in usual activities four to eight weeks postdischarge. Contrary to our data, problems in mobility, self-care, daily activities, and ability to return to work were only identified in approximately half of the participants. In our study, all participants had problems in ADL performance at three months postdischarge, including ability to return to work. These differences could be a reflection of the following: differences in hospital length of stay, with our cases having longer admission days; our sample size was small compared to their 100 inclusions, different ways of testing; in particular, Halpin et al. [9] utilized self-reported outcomes and our study used observational assessment of ADL. Furthermore, our inclusion criteria were patients *with lower ability to perform ADL at discharge* compared to prehospitalization, whereas Halpin et al. [9] included *all* hospital admitted patients diagnosed with COVID-19.

Interestingly, two of the three cases in our study showing significant improvement in ADL performance at follow-up in both motor and process skills were patients needing assistance for personal ADL prior to admission and having coexisting illnesses. Patients with preexisting disabling conditions are more prone to experience physical or psychological effects after COVID-19 [13]. These two cases were observed in easier and much easier ADL tasks during AMPS, e.g., activities like upper body dressing and brushing teeth. They were the only cases observed in the same activities at discharge as well as follow-up. Although the AMPS algorithm takes into consideration the difficulty of tasks, a source of error can occur when participants perform AMPS tasks that are too easy to offer sufficient challenge in identifying difficulties in performance [24]. Raw score skills of the two cases at follow-up indicated sufficient challenge for motor skills, but the AMPS activities chosen may have been too easy to identify difficulties in process skills. Another explanation could be that the cases were more familiar with their test environment. When tested in an inpatient rehabilitation unit of the community, cases had exposure to the community test environment since hospital discharge. Comparatively, other follow-ups were performed on a one-day visit to the hospital where little or no exposure and experience with the hospital test environment was possible. It could be assumed that being tested in unfamiliar surroundings had a negative influence on ADL task performance.

### 4.2. Cognitive Function and Process Skills

Studies have shown that the cut-off score in MoCA of 26 to determine cognitive impairment may be inadequate [28], and some researchers argue cut-offs <25 or even <20, depending on premorbid functional level [28]. Our data cannot provide answers on this subject; however, it is worth noting that our MoCA results are inconsistent with the process ability scores of AMPS. There is conflicting reporting in the literature as to whether higher MoCa scores correlate to a higher functional outcome and ability to perform ADL. Some researchers have found higher MoCA scores related to better functional gains in a general rehabilitation population when using the motor scores of Functional Independence Measure (FIM) compared with MoCA on 116 in-patients on a general rehabilitation unit [33]. In contrast, other researchers [34] have found no statistically significant association between functional performance and MoCA. They used FIM total scores and MoCA to assess functional performance in a sample of 20 participants in an inpatient geriatric hospital setting. In line with this, we found no trends or patterns in higher MoCA scores correlating to higher AMPS scores. AMPS and FIM are, however, not equivalent measures. FIM is used by a multidisciplinary team to assess motor and cognitive items of self-care, transfers, locomotion, communication, social cognition, and sphincter control [34], whereas AMPS is an OT-specific assessment of motor and process skills during activity performance in ADL.

In people diagnosed with stroke, cancer, or cardiac disease, problems of mild cognitive functioning and executive functioning are often not detected on the ward during hospital admission, however, can be detected through ADL testing, including AMPS [35, 36]. Typically, hospital settings are simple and do not match the challenges of real-world settings. In line with this, in our data, two patients had not been referred to OT during admission but were recruited coincidentally through multidisciplinary conferences, where other health professionals described discrepancies between current and pre-COVID-19 ADL performance. Both cases were functional independent prior to hospitalization: one working full time and the other retired. Taking into consideration the cut-off of 1.0 logit in process scores for independent living [24], one would expect these two cases to have a functional habitual level above cut-off and even above risk zone in process logits of 1.3 logit. In both cases, AMPS indicated questionable inefficiency or disorganization during ADL task performance at discharge with no change three months later. The two cases had similar AMPS motor ability measures at both assessments. Higher process skills have been found to be associated with higher cognitive functioning [24]; however, the retiree scored full scores in the cognitive screening of MoCA at both discharge and follow-up, indicating that MoCA may have had a ceiling effect. The other case, with full time employment prehospitalization, showed mild cognitive deficits with a 24 and 25 out of 30 in both MoCA, especially affected in the domain of memory. These cases further depict the lack of pattern between MoCa and AMPS, having very similar AMPS result but different MoCA scores.

### 4.3. Implications for OT Practice and Future Research

The present multiple case study adds to a growing body of evidence on the role of occupational therapists in a hospital setting as part of the initial rehabilitation of patients with COVID-19, as well as postdischarge. Our data describe extensive difficulties in carrying out ADL for this patient population. Occupational therapists can apply performance-based assessments to identify rehabilitation needs of ADL, including possible cognitive rehabilitation needs that may present during ADL performance [35]. This may qualify the initial rehabilitation of patients with COVID-19 and their discharge planning as well as rehabilitation postdischarge as is the case for other patient populations [35]. Guidelines on specific test and intervention methods are yet to emerge [8, 15, 17].

Our findings underline the importance for a comprehensive assessment of COVID-19 patients to identify OT rehabilitation needs. The same methods of testing may not necessarily be relevant to all COVID-19 patients but should include assessment of cognitive functioning and ability to perform ADL.

It is relevant to assess ADL ability of patients with COVID-19, using AMPS in a larger population, preferably in a collaboration with communities for long-term follow-up. Further research could also benefit from investigating which OT assessments best apply to COVID-19 patients during hospitalization and postdischarge, as well as the appropriate timing of testing. Future studies could investigate interventions regarding fatigue and energy management in rehabilitation and the possible connection between fatigue, physical exercise, and cognitive function for this population. The lack of clear patterns between MoCA and AMPS results could indicate a need for further research in adequate assessment for identifying cognitive impairment in COVID-19 patients, including the optimal cut-off in MoCA.

### 4.4. Methodological Considerations and Limitations

The design of the study is a case series, which inherently has some strength and limitations [19, 20]. Case series have methodological limitations in creating causal inferences as there is no control group [19, 20]. Until more solid evidence is available, case series can inform the initial planning of OT interventions with COVID-19 patients and generate hypothesis that can be tested in future analytic studies [19, 20]. One strength of this present study is the triangulation of data sources using standardized tests as well as data from electronic journals providing comprehensive descriptions of the patients. Another strength was author triangulation in relation to the interpretation of findings by experienced researcher [18]. Moreover, it is a strength that follow-up testing could be transferred to community rehabilitation centers when some cases were evidently unable to transport to the hospital for testing [18]. Three cases from three-month follow-up facilitated the opportunity for collaboration between occupational therapists at RH and three different municipalities. It is most likely that these patients would have declined follow-up testing, if testing was not performed in the community. There is great potential in future projects for closer collaboration between hospital and community to assess long-term outcomes after COVID-19, especially for patients with COVID-19 and preexisting disabling conditions. From our experience, these patients want to participate in research projects but prefer participation in their local surroundings as they may be prone to experience further physical or psychological effects after COVID-19 and find transportation to the hospital a burden.

Common to healthcare systems worldwide in 2020, we were learning how to assess and treat patients admitted with COVID-19, on the go. And as such, this study was conducted due to the need for more clinical experience and knowledge about this patient population and how OT can best be provided. There are, however, some limitations due to the nature of planning a study with an unknown long-term trajectory. These limitations include a nonconsecutive and convenience sample. Due to the rapid changes in environment and organization of the new COVID-19 wards, patients were not systematically included or assessed for eligibility. Patients with other primary diagnosis were also included, however, in future research excluding patients not admitted with COVID-19 as their primary diagnoses will make comparisons more adequate. Several patients were lost to follow-up, which reduced the number of participants significantly. It was a limitation that follow-up MoCA was also being used by testers in a separate nonrelated study with a parallel time frame of this current study. A lack of coordination between projects resulted in missing one case at three-month follow-up, and another case had a 60-day gap between AMPS and MoCA.

In addition, we did not know the AMPS ability measures of the cases before admission to hospital, and therefore, we were unable to report exactly how close the patients were to their actual habitual functional AMPS score at follow-up. It was a strength using a comprehensive objective measure of ADL performance in AMPS. This, however, could have been supported by subjective assessments such as the Canadian Occupational Performance Measure (COPM), gaining knowledge on self-perception and satisfaction of occupational performance. As follow-up was performed in different settings with different journal practice, predominant problematic motor and process performance skills were not consequently described in patient journals by the occupational therapist at follow-up.

In conclusion, in a series of eleven hospitalized patients diagnosed with COVID-19 with heterogenic prehospital ADL abilities and various admission trajectories including admission to ICU, the ability to perform ADL was affected at discharge and for the majority at three-month follow-up. Most cases also showed mild cognitive impairment. The comprehensive description of cases and the investigation of similarities and trends adds to the growing academic research on patients with COVID-19 and on how to plan OT intervention during hospitalization and, furthermore, in community rehabilitation units. It also highlights the need for further evidence of the impact of COVID-19 on the ability to perform ADL as well as using occupation-based assessment and treatment in COVID-19 rehabilitation.

## Figures and Tables

**Figure 1:** Study flow diagram.

**Figure 2:** AMPS motor ability measure. Individual AMPS motor ability measures at discharge and 3-month postdischarge in logits. Red horizontal line indicates criterion references cut-off of 2.0 logits, where a person with a score below is likely to begin showing slight clumsiness or physical effort during ADL task performance.

**Figure 3:** AMPS process ability measure. Individual AMPS process ability measures at discharge and 3-month postdischarge in logits. Red horizontal line indicates criterion references cut-off of 1.0 logits, where a person with a score below is likely to begin showing inefficiency and/or disorganization during ADL task performance.

**Figure 4:** MoCA scores. Individual MoCA scores at discharge and 3-month postdischarge. Red horizontal line indicates cut − off score < 26 for mild cognitive impairment.

**Table 1:** Characteristics of participants (*n* = 11).

Age	
Median years (range)	68 (40-87)
Sex	
Male (%)	7 (64)
Employment status	
Employed full time (%)	3 (27)
Unemployed (%)	1 (9)
Retired (%)	6 (55)
Early retirement (%)	1 (9)
Independence in ADL prior to admission	
All ADL (%)	6 (55)
P-ADL (%)	2 (18)
Some P-ADL (%)	3 (27)
Primary diagnose at hospital admission	
COVID-19 (%)	9 (82)
Other diagnose (%)	2 (18)
Patients in ICU (%)	7 (64)
Median days of admission to ICU (range)	24 (10-80)
Days from admission to discharge assessment,	
Median days (range)	20 (7-95)
Isolation for COVID-19 at discharge tests	7 (64)
Discharge destination	
Home with outpatient rehabilitation (%)	5 (45)
Inpatient rehabilitation unit in community (%)	3 (27)
Inpatient rehabilitation unit in community via hospital rehabilitation unit (%)	2 (18)
Rehabilitation unit in hospital, own home, nursing home (%)	1 (9)
Referred to OT	8 (73)
Swallowing assessment (%)	7 (64)
ADL assessment (%)	1 (9)

ADL: activities of daily living; P-ADL: Personal activities of daily living (e.g., washing, eating, and dressing); ICU: intensive care unit; OT: occupational therapy.

**Table 2:** Case descriptions.

Case	Sex age	Civil status	Habitual illness	Habitual functional level	Adm diag	ICU DoA	Referral to OT Initial OT observations	Initial OT treatment goals	OT treatment plan and notes during admission	Days to discharge test^∗^	Iso	Discharge destination ≤ follow − up	Focus of rehabilitation plans (OT and/or PT)
1	M 62	Cohabitating Early retirement	Cardiovascular disease	Mobilizing with a wheeled walker. General weakness, loss of appetite, weight loss. Assistance for medicine administration daily and with bathing every three days. Shower bench and raised toilet seat.	Intra cerebral hemorrhage	19 days	Yes. Swallowing assessment. Moderate dysphagia. Nasogastric tube. Able to hold a glass, but needs physical assistance getting it to the mouth for sips. Cognitive dysfunctions.	To be able to swallow mouth water safely. To be able to keep oral cavity clean from residue independently. To be able to eat texture modified foods and drink thickened liquids.	Reassessment of swallowing. ADL assessment. After 4 days, able to drink moderately thick liquids and eat pureed foods with physical assistance + supplementary nasogastric tube. Facilitation of participation in P-ADL (toothbrushing, washing the face, and lifting a glass to the mouth). Mobilized in a wheelchair and unable to walk. Rehabilitation plan	36	No	Inpatient rehabilitation unit in hospital. Hospital readmission. Initially discharge to own home, but then transferred to a nursing home.	Multidisciplinary neurorehabilitation
2	M 40	Cohabitating Employed full time	None	Independent in all ADL, including work.	COVID-19	43 days	Yes. Swallowing assessment. Able to drink thin liquids and eat pureed foods. Physical assistance in getting food and drink to the mouth, due to lack of strength and coordination of both arms. Difficulty following verbal commands.	To be able to eat minced and moist foods independently.	ADL assessment. Able to brush teeth and dress upper body independently but exhausted by completion. Mobilized in a wheelchair and unable to walk. Rehabilitation plan.	56	No	Inpatient rehabilitation unit in community. Home with outpatient rehabilitation.	Independence in P-ADL and I-ADL. Return to work. Endurance, strength, and manipulation. Swallowing assessment.
3	M 76	Cohabitating Retired	Obesity Cardiovascular lung disease Arthritis	Mobilizing independently in wheelchair. Able to walk short distances with walking frame. Independent in transfers. Independent in some P-ADL, e.g., upper body dressing. Help for I-ADL. Dyspnoea during activity performance. Assistance for medicine dispensing.	Reposition of total knee arthroplasty (TKA)	24 days	Yes. Swallowing assessment. Able to drink small amounts of mildly thick liquids, needing help lifting the cup to the mouth and intermittent verbal prompting to initiate swallow.	To be able to eat pureed foods within seven days. To be able to drink thin liquids within fourteen days.	Reassessments of swallowing. After 6 days, able to drink thin liquids and eat pureed foods, but still being very tired and needing breaks to catch his breath during meals.	77	Yes	Inpatient rehabilitation unit in hospital. Inpatient rehabilitation unit in community.	ADL Transfer methods. Trunk stability. Lower limb exercise after TKA. Upper limb exercise.
4	F 44	Cohabitating Unemployed	Autoimmune disorders Endometriosis	Independent in all ADL, including recent work.	COVID-19	80 days	Yes. Swallowing assessment. Able to drink thin liquids and eat small amounts of minced foods, nasogastric tube. Assistance for positioning in bed. Able to get glass and spoon to her mouth, unable to dress and especially button. Fatigue.	To be able to button clothes. To be able to press down asthma inhaler.	ICU: Reassessment of swallowing. A week after, risk of aspiration, nasogastric tube. Assistance lifting glass and spoon to the mouth. Post-ICU: Re-assessment of swallowing. ADL assessment. Strengthening exercises for the hands. Encourage participation in P-ADL, combining rest with activity to avoid exhaustion. Rehabilitation plan.	95	Yes	Inpatient rehabilitation unit in hospital. Inpatient rehabilitation unit in community. Home with outpatient rehabilitation.	Independence and efficiency during ADL. Return to work. Walking, balance, energy conservation, endurance, strength, and dyspnoea. Pulmonary rehabilitation, including Coping at exhaustion.
5	M 60	Cohabitating Employed full time	Ulcerative colitis	Independent in all ADL, including work.	COVID-19	26 days	No	To be able to shower independently seated within three weeks. To be able to prepare a small meal within two months To be able to walk the dog within four months To be able to mow the lawn within six months To be able to vacuum the house with few breaks within eight months	Project tests. Rehabilitation plan.	39	No	Home with outpatient rehabilitation.	Return to work and complex ADL focusing on endurance, memory and concentration. Pulmonary rehabilitation focusing on endurance, dyspnoea and strength. Mental health and cognition. Energy conservation.
6	F 68	Cohabitating Retired	Hypertension	Independent in all ADL.	COVID-19	Nil	No	To be able to structure everyday life in order to go for walks and regain habitual activities.	Project tests. Rehabilitation plan.	7	Yes	Home with outpatient rehabilitation.	Principles of energy conservation in order to carry out ADL. Strength, pulmonary rehabilitation.
7	M 84	Coliving Retired	Cardiovascular and hematological diseases ataxia	Mobilizing with a wheeled walker. Assistance with showering once a week and support stockings daily. Assistance for I-ADL. Shower bench and raised toilet seat.	COVID-19	Nil	Yes. ADL assessment. Able to brush his teeth when assisted to sitting and with remedies within reach, needing help for most other ADL.	To be able to walk 5-10 meters with a wheeled walker and support of 1 person. To be able to put on a shirt independently within 10 days.	Project tests. Rehabilitation plan.	17	Yes	Inpatient rehabilitation unit in community.	Independence in P-ADL and mobilizing with wheeled walker. Endurance.
8	F 57	Cohabitating Employed full time	Hypertension Obesity	Independent in all ADL, including work.	COVID-19	10 days	Yes. Swallowing assessment. Able to drink thin liquids and eat minced foods, nasogastric tube.	To be able to eat normal foods. To be able to eat and drink sufficiently, not needing supplementary feeding. To be able to shower sitting, remedies within reach in 5 days.	Reassessment of swallowing. ADL assessment. After 6 days, able to eat and drink sufficiently and eat normal foods. Rehabilitation plan.	15	Yes	Home with outpatient rehabilitation. Hospital readmission.	Efficient and independent complex ADL focusing on motor ability skills and upper extremity. Walking. Strength, endurance, and dyspnoea.
9	M 87	Cohabitating Retired	Malignant melanoma	Mobilizing with a wheeled walker. Independent in P-ADL. Assistance with I-ADL.	COVID-19	Nil	Yes. Swallowing assessment. Weakness, dysphagia, low energy for chewing. Able to eat minced foods and drink mildly thick liquids. Assistance to complete all P-ADL.	To be able to drink thin liquids To be able to eat soft foods To be able to wash his face with a face cloth independently, within 7 days.	Reassessment of swallowing. ADL assessment. Facilitation of participation in P-ADL (eating, drinking, toothbrushing, and washing the face). Rehabilitation plan.	19	No	Local hospital. Inpatient rehabilitation unit in community. Death	Independence in P-ADL focusing on strength in upper extremity. Energy conservation and pulmonary rehabilitation. Sit–stand, coordination swallow, and breath.
10	F 79	Living alone Retired	None	Independent in all ADL, except heavy shopping.	COVID-19	10 days	Yes. Swallowing assessment. Aspiration of thin liquids and pain during swallowing. Pureed foods and moderately thick liquids + nasogastric tube.	To be able to drink mildly thickened liquids and soft foods within 7 days.	Reassessment of swallowing. After 4 days, able to drink thin liquids and eat soft foods. Rehabilitation plan.	20	Yes	Home with outpatient rehabilitation.	Complex ADL, like leisure activities, focusing on endurance, and process ability skills.
11	M 86	Cohabitating Retired	Cardiovascular disease. Chronic kidney disease. Dialysis. Diabetes.	Mobilizing with a wheeled walker. Assistance for support stockings daily. Independent in all other P-ADL. Participate in some I-ADL like shopping.	COVID-19	Nil	No	To be able to shower independently as prehospitalization.	Project tests. Rehabilitation plan.	19	Yes	Home with outpatient rehabilitation.	ADL focusing on strength, manipulation, coordination of the upper extremity, energy conservation, and dyspnoea. Cognition focusing on visuospatial/executive domains and memory. Strength, endurance, balance, and walking. Sit-stand.

Adm diag: admission diagnosis; ICU: intensive care unit; DoA: days of admission; OT: occupational therapist. ^∗^Days from admission to discharge test at Rigshospitalet. Iso: isolation at discharge test; PT: physiotherapist; rehabilitation plan: referral for further community rehabilitation; M: male; F: female; P-ADL: personal activities of daily living (e.g., washing, eating, and dressing); I-ADL: instrumental activities of daily living (e.g., work, cooking, and shopping).

**Table 3:** Difficulty of AMPS activities across cases.

	At discharge, *n* = 22^∗^	At follow-up, *n* = 18^∗^
Much easier than average ADL tasks (logit challenge: 0.7, 0.5), e.g., upper body dressing-garment within reach	11 (50)	5 (28)
Easier than average ADL tasks (logit challenge: 0.4, -0.2), e.g., upper body grooming/bathing	8 (36)	2 (11)
Average ADL tasks (logit challenge: 0.1, -0.1), e.g., changing sheets	3 (14)	6 (33)
Harder than average ADL tasks (logit challenge: -0.2, -0.4), e.g., pasta with sauce and beverage—two persons		3 (17)
Much harder than average ADL tasks (logit challenge: -0.5, -0.7), e.g., scrambled/fried eggs, toast, and coffee/tea—one person		2 (11)

*n* (%). ^∗^2 AMPS activities must be carried out per test.

**Table 4:** AMPS activities performed and difficulty of activities. AMPS and MoCA results at discharge and follow-up.

Case	AMPS activity discharge	AMPS activity follow-up	Chal log dish	Chal log FU	Result logit discharge	Result logit follow-up	Percentile rank at discharge	Percentile rank at follow-up	MoCA discharge	MoCA follow-up
1	Upper body grooming/bathing	¤	0.2		M -1.0		<1		8/30	¤
	Upper body dressing-garment within reach		0.7		P 0.0		<1			
2	Brushing teeth	Boiled egg(s) served in cup(s)	0.6	-0.1	M 0.7	M 1.5	<1	1.1	18/30	29/30
	Upper body dressing-garment within reach	Coffee/tea and cookies served on a tray-2/3 persons	0.7	-0.1	P 0.9	P 1.1	3.5	9.5		
3	Upper body grooming/bathing	Upper body grooming/bathing	0.2	0.2	M -0.6	M 0.7	<1	<1	20/30	23/30
	Upper body dressing-garment within reach	Upper body dressing-garment within reach	0.7	0.7	P 0.3	P 1.0	<1	21.1		
4	Upper body grooming/bathing	Pasta with sauce and beverage-two persons	0.2	-0.4	M 0.1	M 1.6	<1	2.3	26/30	¤
	Upper body dressing-garment within reach	Hand washing, drying, and putting away dishes	0.7	0.0	P 0.9	P 1.6	3.5	50.0		
5	Upper body dressing-garment within reach	Scrambled/fried eggs, toast, and coffee/tea-one person	0.7	-0.5	M 1.2	M 2.3	<1	61.9	24/30	25/30
	Changing sheets and “duvet” cover on a freestanding bed	Fresh fruit salad-2 persons	0.0	-0.3	P 1.2	P 1.0	21.1	9.5		
6	Showering	Coffee/tea and cookies served on a tray-2/3 persons	0.1	-0.1	M 1.3	M 2.4	2.3	78.9	30/30	30/30
	Upper and lower body dressing-garments stored	Putting away clean dishes from a dishwasher	0.2	0.0	P 1.2	P 1.0	21.1	9.5		
7	Brushing teeth	Brushing teeth	0.6	0.6	M -0.5	M 0.8	<1	1.1	24/30	21/30
	Washing and drying the face	Washing and drying the face	0.5	0.5	P 0.8	P 1.7	9.5	84.2		
8	Showering	Scrambled or fried eggs, toast, and brewed coffee or tea-one person	0.1	-0.5	M 0.7	M 1.1	<1	<1	28/30	¤
	Upper and lower body dressing-garments set out	Changing sheets and “duvet” cover on a freestanding bed	0.4	0.0	P 1.7	P 1.3	61.9	21.1		
9	Brushing teeth	¤	0.6	¤	M -1.3	¤	<1	¤	16/30	¤
	Brushing or combing hair		0.9		P 0.8		9.5			
10	Changing sheets and “duvet” cover on a freestanding bed	¤	0.0	¤	M 1.9	¤	61.9	¤	24/30	¤
	Upper and lower body dressing-garments set out		0.4		P 1.8		90.5			
11	Upper body grooming/bathing	Ironing multiple garments and putting garments away	0.2	-0.2	M 0.5	M 0.6	<1	<1	17/30	22/30
	Upper body dressing-garment within reach	Pot of brewed coffee-one or two persons	0.7	0.0	P 0.9	P 1.2	15.8	38.1		

Chal log dish: challenge in logits at discharge; Chal log FU: challenge in logits at follow-up; percentile rank: percentage of people with lower AMPS measures; M: motor ability measure expressed in logits; P: process ability measure expressed in logits; ¤: missing.

**Table 5:** MoCA domain scores (*n* = 11).

Case	Education years	MoCA score at hospital discharge						MoCA score at 3-month follow-up					
		Attention (0-6)	Visuospatial abilities (0-4)	Executive functioning (0-4)	Memory (0-5)	Language (0-5)	Orientation (0-6)	Attention (0-6)	Visuospatial abilities (0-4)	Executive functioning (0-4)	Memory (0-5)	Language (0-5)	Orientation (0-6)
1	+12	1	1	0	1	4	1	¤	¤	¤	¤	¤	¤
2	-12	5	2	0	0	4	6	5	3	4	4	5	6
3	+12	2	3	2	3	4	6	5	3	3	2	5	5
4	+12	5	4	2	5	4	6	¤	¤	¤	¤	¤	¤
5	+12	6	3	3	1	5	6	5	3	3	3	5	6
6	+12	6	4	4	5	5	6	6	4	4	5	5	6
7	-12	6	2	2	4	4	5	3	2	2	2	5	6
8	+12	6	4	3	5	5	5	¤	¤	¤	¤	¤	¤
9	+12	4	2	0	0	4	6	¤	¤	¤	¤	¤	¤
10	-12	4	1	3	4	5	6	¤	¤	¤	¤	¤	¤
11	+12	5	1	1	0	4	6	6	2	2	3	3	6

Higher numbers = higher cognitive function; ¤: missing data.

## Data Availability

Statistical analysis plan and deidentified data can be available upon reasonable request to the corresponding author.
